# Classification and Pathological Diagnosis of Idiopathic Interstitial Pneumonia

This article has been retracted.

**DOI:** 10.1155/2022/1198581

**Published:** 2022-05-31

**Authors:** Zhihua Chen, Wenqiang Huang, Yibo Song

**Affiliations:** Department of Pulmonary and Critical Care Medicine, Maoming People's Hospital, Maoming, Guangdong 525000, China

## Abstract

Idiopathic interstitial pneumonia (IIP) is a group of progressive lower respiratory tract diseases of unknown origin characterized by diffuse alveolitis and alveolar structural disorders leading to pulmonary fibrillation and hypertension, pulmonary heart disease, and right heart failure due to pulmonary fibrosis, and more than half of them die from respiratory failure. To address these problems of overly complex prediction methods and large data sets involved in the prediction process of interstitial pneumonia, this paper proposes a prediction model for interstitial pneumonia which is based on the Gaussian Parsimonious Bayes algorithm. Three usual tests of pneumonia, specifically from various patients, were collected as the sample set. These samples are divided into training and testing sets. Additionally, a cross-validation strategy was used to avoid the overfitting problem. The results showed that the prediction model based on the Gaussian Parsimonious Bayes algorithm predicted 92% accuracy on the test set, and the Parsimonious Bayes method could directly predict the final detection of interstitial pneumonia based on the usual pneumonia test pneumonia. In addition, it was found that the closer the data distribution of the sample set was to a normal distribution, the higher the prediction accuracy was, and then, after excluding pneumonia from the test below 60 points, the prediction accuracy reached 96%.

## 1. Introduction

In 1969, Liebow first proposed a group of five classical pathological histological types of diffuse interstitial pneumonia of unknown origin, namely, universal interstitial pneumonia (UIP), desquamation interstitial pneumonia (DIP), bronchiolitis obliterates with interstitial pneumonia (BIP), occlusive bronchitis obliterates with interstitial pneumonia (IIP), lymphocytic interstitial pneumonia (LIP), and giant cell interstitial pneumonia (GIP) [1]. Over the next 30 years, the classification has changed, with the concept of BIP being replaced by bronchiolitis obliterans organizing pneumonia (BOOP), and giant cell interstitial pneumonia being eliminated because of its association with heavy metal. In 1998, Larsen and Colby renamed this diffuse interstitial lung disease as idiopathic pulmonary fibrosis (IPF) and reintroduced five new pathological types in addition to UIP, including DIP aspiration bronchitis with interstitial lung disease (respiratory bronchiolitis). In addition to UIP, five new pathological types have been reintroduced, including DIP aspiration bronchitis with interstitial lung disease (RBILD), acute interstitial pneumonia (AIP) or Hamman–Rich syndrome, and nonspecific interstitial pneumonia (NSIP) [2]. The three types of LIP, GIP, and BOOP were excluded from the IIP family because LIP was found to be a lymphoproliferative disorder associated with immune deficiency and GIP was a manifestation of heavy metal pneumoconiosis.

In recent years, the study of interstitial pneumonia prediction has become the focus of researchers, and predicting end-of-course pneumonia in advance by reasonable means will help attending physicians to implement targeted teaching. Additionally, it will help interstitial pneumonia with learning difficulties and improve interstitial pneumonia with excellent learning pneumonia.

Due to the development of online learning, there have been new developments in research on interstitial pneumonia prediction such as pneumonia prediction that is based on interstitial pneumonia learning behaviors in online course learning [3]. Likewise, pneumonia prediction is based on the comparison of the advantages and disadvantages of various classification algorithms considering the learning background of online learners, their home environment, and the behavioral characteristics of learners [2, 3]. The second is the research on pneumonia prediction based on independent algorithm or fusion of multiple algorithms, such as the research on pneumonia prediction based on Bayesian algorithm, which is mainly through parameter learning through network structure and finally applied to the prediction of interstitial pneumonia. In the paper “pneumonia prediction based on fuzzy clustering and support vector regression,” Zuo jun calculated the similarity of each pneumonia on the basis of constructing the pneumonia map, combined with the prediction method of collaborative filtering interstitial pneumonia and the prediction of interstitial pneumonia based on multiple regression and decision tree model.

In 2000, the ATS and ERS published a comprehensive multinational expert opinion on the diagnosis and treatment of IPF, which provided a new international consensus on the classification and diagnosis of IPF, and the committee concluded that UIP is a histopathological category consistent with IPF, and therefore, IPF refers specifically to UIP, while DIP, RBILD, NSIP, and AIP are separate disease entities that belong to the same category as UIP/IPF. The IPF refers specifically to UIP, while DIP, RBILD, NSIP, and AIP are distinct disease entities that, together with UIP/IPF, belong to the idiopathic interstitial pneumonia (IIP), the ATS/ERS category of the IIP in 2000. Two years later, in 2002 [8], the ATS published a revision of the ATS/ERS classification, redefining the subtypes of IIP to include not only UIP/IPF, NSIP, DIP, RBILD, and AIP but also idiopathic LIP and cryptogenic organizing pneumonia (COP). COP is the same concept as idiopathic BOOP (IBOOP). The new ATS/ERS classification unifies the different views and perceptions of the concept and classification of IIP in the past pathology and clinical practice and facilitates the diagnosis and treatment of IIP as well as international research cooperation. Of course, the applicability and rationality of this classification have yet to be tested and refined in practice.

The ATS/ERS classification also points out that the diagnosis of each type of IIP depends on VATS/open lung biopsy in addition to clinical and imaging data, but the final pathological diagnosis should be closely linked to clinical data and imaging, that is, the clinical-radiologic-pathologic diagnosis (CRP diagnosis). The diagnosis by clinicians, radiologists, or pathologists alone may be one-sided, and a CRP diagnosis should be performed whenever possible. For a long time, different classification criteria and terminology have been used in pathology and clinical practice resulting in a confusing nomenclature of the various subtypes of IIP, which is not conducive to diagnosis and treatment [7].

The plain Bayesian algorithm is simple to use and works well in various types of studies, and it appears in a large number of studies, for example, research on text classification based on the plain Bayesian approach [9], research on semantic annotation combining the plain Bayesian algorithm with Bootstrapping method [10], and research on improving the plain Bayesian algorithm and applying it to intrusion detection [11]. In addition, good suggestions have been shown in combination with other algorithms for application [3, 11–13].

In this study, the data collection for interstitial pneumonia prediction was limited to a particular course, which reduced the difficulty of the data collection process, using the plain Bayesian method. The prediction results were constantly revised using empirical knowledge and thus ensuring that these results were more closely evaluated objectively. In conclusion, the diagnosis and classification of HP are among the new problems for pathologists. These are responsible to carefully review the film and closely correlate clinical and imaging data for ensuring a correct diagnosis. Although all types of HP show varying degrees of interstitial inflammation and fibrosis, each type has its own lesion characteristics. In terms of lesion progression, all types show lesions at the same stage, except for UIP, which shows inconsistent progression (i.e., intermingling of old and new lesions and near-normal lung tissue between lesions). DIP is mainly characterized by diffuse intra-alveolar macrophage accumulation, while RBILD has similar pathological changes to DIP, except that the lesions are relatively confined to the respiratory [13]. Pathological changes of RBILD are similar to those of DIP, except that the lesions are relatively confined to the respiratory bronchi and their surrounding air space, with a distinctive respiratory bronchiectasis. The foci of fibrinolysis cells are mainly seen in UIP, with hyaline membrane formation in AIP, but not in the other types.

The remaining sections are arranged as follows: the plain Bayesian approach is described in detail in Section 2 where a Section 2.1 is dedicated to Bayes' theorem and its explanation as it is the foundation of the proposed study. Additionally, pathological changes and pathological diagnosis of each HP type are presented in Section 2.4. Results and observations, which are collected through various experiments, are presented in Section 3. Finally, a generalized discussion section along with an extensive summary of the proposed work is presented in Section 4 to conclude the paper.

## 2. Plain Bayesian Approach

The Naive Bayes method is a classification method that is based on Bayes' theorem, a well-known approach, and the assumption of conditional independence of features. For a given training dataset, the joint input/output probability distribution is first learned which is based on the feature conditional independence assumption, and then, the posterior probability of the given input *x* is maximized by using Bayes' theorem to find the output *Y*.

### 2.1. Bayes' Theorem

Let *A*_*i*_ (1 ≤ *i* ≤ *n*) events satisfy the following conditions:

(1) Two are mutually incompatible, that is, when *i* = *j*, there is *A*_*i*_∩*A*_*j*_=∅
(2) P(*A*_*i*_) > 0(1 ≤ *i* ≤ *n*)
(3) Sample space Ω=∪_*i*=1_^*n*^*A*_*i*_
(4) Then, for any event *B*, the following equation holds:
  (1) $$\begin{array}{c} P\left(A_{i}|B\right)=\frac{P\left(A_{i}\right)\times P\left(B|A_{i}\right)}{\sum_{i=1}^{n}P\left(A_{i}\right)\times P\left(B|A_{i}\right)},i=1,2\cdots \cdots n, \end{array}$$
   where *P*(*A*_*i*_*|B*) is the probability that event *B* will occur given the occurrence of the event *A*_*i*_, also known as the “likelihood value,” and is not the probability density.

### 2.2. Plain Bayesian Formula

Let *B*_*j*_(1 ≤ *j* ≤ *m*) events satisfy the following conditions:

(1) Two are independent of each other; that is, when *i* ≠ *j*, there are *P*(*B*_*i*_*|B*_*j*_)=*P*(*B*_*i*_) or *P*(*B*_*j*_*|B*_*i*_)=*P*(*B*_*j*_)
(2) *P*(*B*_*j*_) > (1 ≤ *j* ≤ *m*). The following equation holds:
  (2) $$\begin{array}{c} \text{P}\left(A_{i}|B_{1}B_{2}\ldots \ldots B_{m}\right)=\frac{\text{P}\left(A_{i}\right)\times \prod_{j=1}^{m}P\left(B_{j}|A_{i}\right)}{\sum_{i=1}^{n}P\left(A_{i}\right)\times \prod_{j=1}^{m}P\left(B_{j}|A_{i}\right)},i=1,2\cdots \cdots n. \end{array}$$

Since the denominator in equation (2) is a fixed value, only the numerator part can be calculated for classification. The plain Bayes formula is applied to prediction, that is, given a specific input *B*_*j*_(1 ≤ *j* ≤ *m*), the joint probability distribution of each *A*_*i*_(1 ≤ *i* ≤ *n*) and *B*_*j*_(1 ≤ *j* ≤ *m*) is calculated, and the maximum of the *n* values is used as the prediction result for the specific input value.

### 2.3. Gaussian Parsimonious Bayesian Classifier

Generally, there are three commonly used models for the plain Bayesian algorithm: (1) Gaussian model, (2) polynomial model, and (3) Bernoulli model. Bernoulli model, like a polynomial model, is applicable to the case of discrete features. The difference is that the methods of calculating prior probabilities and class probabilities are different. Gaussian model is adapted to deal with continuous feature variables. Gaussian model assumes that each dimensional feature data obey normal distribution and what needs to be calculated is the mean and variance of each dimensional feature to calculate its probability density value from each dimensional feature value. This value is also known as the likely value [9].

For the specific problem of pneumonia prediction, in the plain Bayesian formulation, *B*_*j*_ is assumed to be a continuous-valued attribute and obeys a Gaussian distribution. It is assumed that P(B_j_*|*A_i_) ~ *N*(*μ*_A_i_,j_, *σ*_A_i_j_^2^), where *μ*_A_i_,j_ and *σ*_*A*_*i*_*j*_^2^ are the mean and variance of the values taken by the *A*_*i*_th class of samples on the jth attribute, respectively.

Then, the probability density function of *P*(*B*_*j*_*|A*_*i*_) is

(3) $$\begin{array}{c} P\left(B_{j}|A_{i}\right)=\frac{1}{\sqrt{2\pi }\sigma_{A_{i}}}\exp\left(-\frac{{\left(B_{j}-\mu_{A_{i}}\right)}^{2}}{2\sigma_{A_{i}j}^{2}}\right). \end{array}$$

The Gaussian Parsimonious Bayesian classifier is obtained as follows:

(4) $$\begin{array}{c} h_{nb}\left(\text{B}\right)=\arg\max_{A_{i}\in y}\text{P}\left(A_{i}\right)\times \prod_{j=1}^{m}P\left(B_{j}|A_{i}\right), \end{array}$$

where the input values *B*=(*B*_1_, *B*_2_,…, *B*_*m*_), *P*(*A*_*i*_) are the prior probabilities of the *A*_*i*_rd class of samples, and *h*_*nb*_(*B*) represents the predicted outcome of the input values.

### 2.4. Pathological Changes and Pathological Diagnosis of Each HP Type

1. UIP/IFP: UIP is the most common form of IIP (about 65%), and its exact incidence is not known, estimated to be about (3–6)/100,000 people, with a poor response to glucocorticoids and a poor prognosis. The clinical manifestations are dry cough and dyspnea, and inspiratory sounds can be heard in more than 80% of patients, most notably at the base of both lungs. Pulmonary abnormalities are mainly moderate to severe restrictive ventilatory and/or diffusion dysfunction. Laboratory tests are unremarkable, with some patients (10%–25%) having positive serum antinuclear antibodies (ANA) and rheumatoid factors (RF). The chest radiograph mainly shows reticular shadows at the base and periphery of both lungs, often bilateral and asymmetric, with reduced lung volumes. High-resolution CT is important for the diagnosis of UIP, which mainly shows lamellar, mainly basal, reticular shadows in both lungs, and may have a small amount of hair glass shadow. The pathology of UIP is characterized by inconsistent progression of lesions, interstitial inflammation, fibrosis, and honeycomb changes. Visual observation: both lungs are reduced in size, increased in weight, harder in texture, focal scar formation in the dirty pleura, and emphysema or even alveolar formation is seen. The section showed diffuse solid areas in both lungs, with varying severity, and the severely affected areas formed multiroom cystic structures, that is, honeycomb lung [10]. On low magnification: the lesions were patchy, mainly involving the suppliers and lung parenchyma, with interstitial inflammation, fibrosis, and honeycomb changes, varying in severity, with a mixed distribution of old and new lesions, and normal lung tissue visible between the lesions. The early lesions are widened and congested alveolar septa, infiltrated by lymphocytes, plasma cells, histiocytes, and scattered neutrophils, and accompanied by type II alveolar epithelium and fine bronchial epithelial hyperplasia, with macrophages visible in some alveoli; the fibrous areas have varying amounts of collagen fibers deposited, with relatively few inflammatory cells, and the alveolar interstitial capillary beds are reduced or even completely disappeared, with pseudoscience structures forming between them, covered with hyperplastic type II alveolar epithelium. The alveolar epithelium is covered with hyperplastic type II alveolar epithelium. The area of the cellular lung is composed of cystic fibrous air spaces of varying sizes covered with fine bronchial epithelial cells. In the fibrous and cellular lung areas, respiratory airways, alveolar ducts, and reconstructed walls were found to be heavily lined with hyperplastic smooth muscle, forming what is known as “mysterious.” In addition to the old foci (scar foci with collagen deposition) mentioned above, there are also fibroblast foci, which are composed of a large number of fibroblasts with a background of mucus matrix, located in the interstitial lung and protruding towards the luminal surface of the overlying respiratory epithelium. In conclusion, fibroblast foci, scarring with collagen deposition, the coexistence of different contemporaneous lesions and focal lesions are important in the diagnosis of UIP and are also important in differentiating it from other types of HP [11].
2. NSIP: in 1994, the concept of NSP was first introduced by Katzenstein and Fiorilli9 especially for those cases of unclassifiable interrogative pneumonia which were pathologically histologically distinct from UIP, DIP, BOOP, LIP, and GIP. Subsequent studies have shown that NSIP is not a garbage can combined and that this group of cases has similar clinical and pathologic manifestations and should be treated as a separate pathologic entity. 2000 and 2002 ATS/ERS classifications both recognized the status of idiopathic NSTP in the HP family [36]. However, it was also noted that due to the short period of time in which NSIP has been recognized, there is a need for the onset of NSIP is predominantly in middle-aged and elderly patients but can occur in children with a mean age of 49 years, with an insidious or subacute onset, and its etiology is unclear. The main clinical manifestation is progressive dyspnea and cough. High-resolution CT shows symmetrical hairy glass shadow in both lungs or solid shadow in the alveolar space of both lungs [11]. Compared with UIP, most patients with NSIP have a better response to corticosteroids and a relatively good prognosis, with a 5-year mortality rate of 15% to 20%. The uncommon pathological features of NSIP can be summarized as varying degrees of interstitial inflammation and fibrosis in the lung. According to the number of interstitial inflammatory cells and the degree of fibrosis, Katzenstein and Fiorilli classified NsP into three different types: (i) cell-rich type: it accounts for about 50% of cases, mainly manifests as interstitial inflammation with little or almost no fibrosis and is characterized by a mixed infiltration of chronic inflammatory cells, mainly lymphocytes and plasma cells, in the alveolar septum, and its inflammatory cell infiltration is the degree of inflammatory cell infiltration, which is more prominent than in other types of interstitial lung disease such as UIP and DIP. In contrast to LIP, there is no significant destruction of alveolar structure, and the number of plasma cell infiltrates is more prominent in this type. Interstitial inflammation is often accompanied by hyperplasia of the alveolar respiratory epithelium. (ii) The mixed type (Figure 1 in about 40% of cases) has a large number of chronic inflammatory cell infiltrates and marked collagen fibrillation in the interstitial. This type is not easily distinguished from UIP, and the main point of differentiation is that the lesions are relatively uniform throughout the lung, without honeycomb lung, and some fibroblast foci are seen, but the number is small. (iii) Fibrosis type accounts for about 10% of cases, in which the interstitial lung is dominated by dense collagen fiber deposits with a mild inflammatory response or lack of inflammation. Focal foci of fibrous sequestration cells (lack of active fibrosis) are rarely present, and the consistency of the lesions is a key differentiator from UIP. Small focal BOOP-like lesions may be present in about half of the patients with NSIP, but they are small and inconspicuous and do not exceed 10% of the total lesions.
3. DIP: Liebow and Carrington first introduced the concept of DIP by naming the cells gathered in the alveoli as detached alveolar epithelium, and subsequent studies found that the cells gathered in the lumen of these alveoli were mainly macrophages rather than alveolar epithelial cells, and the concept of “detached” was inaccurate, but now the name has been used. The treatment and prognosis of DIP are better than UIP, with a 10-year survival rate of about 70%. DIP is most common in smokers, with an average age of onset of 42 years. Half of the patients have pestle finger. Pulmonary function is restrictive, by reducing diffusion and hypoxemia. General laboratory tests are unremarkable. 20% of patients have nearly normal chest radiographs. In approximately one-quarter of patients, chest radiographs and high-resolution CT scans show diffuse gross glassy changes in the middle and lower lung fields, and later linear reticular and nodular interstitial images [3]. Lung biopsies show diffuse intra-alveolar macrophage aggregates that uniformly distribute. These changes are particularly pronounced around the respiratory fine bronchi and diffuse into the distal air spaces and even throughout the lung parenchyma. In addition to mild to moderate thickening of the alveolar wall, there is no fibrosis scarring, cellular lung, absent or inconspicuous fibroblastic foci, and proliferating fibrous tissue showing at the same stage. Inflammation in the interstitial was mild in extent and degree and consisted mainly of lymphocytes as well as a small number of plasma cells (Figure 2).
4. RBD: in 1987, Myers et al., “first reported 6 cases of RBILD, described as a large accumulation of pigmented macrophages in the respiratory fine bronchi and surrounding air space, which is very similar to DP. In addition, it is not easily distinguishable from DIP in terms of the patient population, response to treatment, disease course, and prognosis. The average age of onset of RBILD is 36 years, with slightly more males than females, and all cases reported to date have a history of smoking; the clinical presentation is similar to that of DP, with rare pestle-like fingers (toes) and popping sounds in both lungs. High-resolution CT scans in about 2/3 of patients show ridiculous shadows and a lack of hairy glass-like changes. The pathological changes of RBD are similar to those of DIP, except that the disease is relatively confined to the respiratory bronchioles and their surrounding air spaces, which have a large number of pigmented macrophage aggregates, but the distal air spaces are not involved, and there is obvious respiratory bronchitis, alveolar septal thickening, and epithelial hyperplasia similar to those of DIP (Figure 3).
5. AIP: it is the most common form of fulminant lung injury, with a mean age of onset of 49 years” and no significant gender difference. The onset of the disease is rapid (within days to weeks), with fever, cough, and shortness of breath followed by respiratory failure, and no specificity in routine laboratory tests. X-ray chest radiographs show diffuse, bilateral lung shadows, and CT scans show bilateral symmetrical patchy hairy glass shadows. The diagnosis of AIP requires a clinical presentation of idiopathic AHDS of unknown origin. The pathological features of the disease are consistent with the lesion, the alveolar septum is widened significantly, there are oval to spindle-shaped fibroblasts and scattered lymphocytes and plasma cells infiltrate, the alveolar type II cistern is proliferated, the fine bronchial epithelium may have squamous epithelial growth, and the alveolar septum is widened significantly area can be seen in the size of the alveolar lumen. A small amount of hyaline membrane was present in a few alveolar lumens (Figure 3). This is the key point of differentiation from other HP. Very few patients can survive with timely and correct treatment, and the lungs can return to normal or progress to end-stage cellular fibrosis.
6. COP: it is a clinicopathologic entity first proposed by Davison et al in 1983, referring to mechanized pneumonia of unknown cause, the same concept as BOOP of unknown cause (i.e., idiopathic BOOP), and the 2002 AIS/ERS classification does not include BOOP of known cause (secondary BOOP). The age of onset of COP is 50–60 years old, with a mean age of 55 years, without gender differences, and is not associated with smoking. The duration of the disease is usually within 2–6 months, and 2/5 of patients have flu-like symptoms such as cough, fever, malaise, malaise, and weight loss. There is often a popping sound at the end of inspiration. Routine laboratory tests are not specific. Pulmonary function is mainly characterized by restrictive ventilation impairment, and hypoxemia at rest and after exercise is a common feature. The chest radiograph showed bilateral diffuse alveolar shadow with normal lung volumes, recurrent and wandering shadows were common, and unilateral alveolar shadow was rare. High-resolution CT shows patchy intra-alveolar solidity, hairy glass shadows, small nodular shadows, and thickening and dilatation of the bronchial walls, mainly in the peri-pulmonary area, especially in the lower lung fields [12]. 2/3 of patients have a good response to corticosteroids. The main pathological changes are organic pneumonia in the small airways and alveolar lumen of the respiratory fine bronchi and below. The lesions are monochromatic, consistent in phase, patchy, and peribronchial in distribution, and located in the air space without destruction of lung structures.
7. IP: Liebow and Carrington used the term “lymphocytic interstitial pneumonia” in 1969 to describe a species of interstitial pneumonia different from LPDP, BP, and GP, but later found that LIP was actually a group of pulmonary lymphoid proliferative diseases and was removed from the HP family. The 2002 ATS/ERS classification reclassified idiopathic LIP into the HP family mainly because of the need to consider LIP in the differential diagnosis of HP and because it is an unexplained interstitial pneumonia in its own right. It is relatively common in people with HV infection, other immunodeficiencies, and autoimmune diseases and is associated with Sjogren's syndrome in 1/3 of patients. Pathologically, it is characterized by diffuse infiltration of lymphocytes, plasma cells, and histiocytes in the interstitial, especially in the alveolar septa (Figure 4), with hyperplasia of type II alveolar epithelium and an increase in macrophages in the alveolar space, often with the formation of lymphoid follicles along the lymphatic vessels with only a germinal center. Alveolar structural alterations and narcotizing granuloma formation were sometimes seen, but narcotizing granulomas and more Dutch vesicles (PAS-positive spherical inclusion in the nucleus) were absent, and intra-alveolar mechanization and phagocytic aggregation were rare or mild. Immunoglobulin light chain staining revealed polygonal B cells. The differential diagnosis includes bronchial mucosa-associated lymphoid hyperplasia (diffuse lymphoid hyperplasia), nodular lymphoid hyperplasia, and malt- and small-cell lymphoma, as well as NSTP, allergic pneumonia, and UIP. Evidence in support of lymphoma is the immaturity of the infiltrating cells, the presence of infiltration of bronchial cartilage, vessel walls, and dirty pleura, and the distribution of infiltrating lesions along lymphatic vessels. Immunohistochemistry and gene rearrangement tests help to identify.

## 3. Experiments for Pneumonia Prediction

### 3.1. Experimental Analysis

The experiments in this paper were programmed in Python, and the data set was stored in an Excel table. Through the experiments, it was found that the Gaussian Bayesian classifier had good results for interstitial pneumonia prediction, and the sample set included a total of 465 records. Among them, the training data consisted of 348 records, the prediction data consisted of 117 sample records, and the classification accuracy reached 92%, and the experimental results are shown in Table 1.

When all pneumonia scores below 60 in the three tests were excluded again, the sample set consisted of 408 records in total. Among them, the training data consisted of 306 records, and the prediction data consisted of 102 sample records, with a classification accuracy of 96%, and the experimental results are shown in Table 2.

### 3.2. Data Model

In general, ideally, the interstitial pneumonia test pneumonia should satisfy a normal distribution, but from the collected data, all three tests of interstitial pneumonia showed a negatively skewed distribution, as shown in Figure 5. In order to verify whether the original data set satisfies the normal distribution of the prediction results, this paper will eliminate the data with a large degree of deviation at both ends, and the normal distribution graph after eliminating the data with less than 60 points is shown in Figure 6. The comparison between Figures 1, 2 and 6 shows that after eliminating the pneumonia with less than 60 points again, the interstitial pneumonia test pneumonia is more concentrated and more close to the fitted normal distribution graph (the thinnest line of graphs in Figure 6). Therefore, as inferred from the Gaussian Parsimonious Bayes classifier, after further exclusion of pneumonia below 60 points, it should be able to better predict pneumonia at the end of the interstitial pneumonia period results.

### 3.3. Comparison of Experimental Methods

The Gaussian Bayesian algorithm is a generative model, while the generative model models the posterior probabilities, tries to describe the joint distribution of *x* and *y*, and estimates the joint probability distribution *P*(*x*), *y*. Support vector machine classification algorithms, on the other hand, are discriminative models. In a basic machine learning problem, there are usually two components, input and output; for example, for classification, the discriminative model seeks the optimal classification surface between different classes and estimates the conditional probability distribution *P*(*y|x*).

Support vector machine is an excellent classification algorithm for the purpose of obtaining good statistical laws with a small statistical sample size. Depending on the specific problem, some data are linearly separable and some are not, and different kernel functions need to be chosen for testing. As we know that the support vector machine algorithm does not emphasize the normality of the feature dataset, it is not necessary to remove pneumonia below 60 points to ensure the normality of the data but to directly process all samples including a total of 465 records and the predicted data including 117 sample records. In addition, based on the preprocessing of pneumonia grade markers for the data samples, the linear kernel function is selected for the test. Experimental results show that the classification accuracy reached 99%, and the experimental results are shown in Table 3.

## 4. Conclusion

Although the plain Bayesian algorithm needs to satisfy the assumptions of feature independence and feature equivalence, it is still an excellent classification algorithm that is successfully applied to document classification. Considering that the Bayesian approach is characterized by combining prior and posterior probabilities, that is, it avoids the subjective bias of using only prior probabilities and the overfitting phenomenon of using sample information alone. In this paper, this algorithm is combined with the assumption that interstitial pneumonia may satisfy a normal distribution, that is, the Gaussian Parsimonious Bayes algorithm is applied to interstitial pneumonia prediction, and good results are obtained. The results found that the closer the sample data are in the normal distribution, the better the algorithm's prediction is, but it is slightly less effective than the classification effect of the support vector machine algorithm. Some articles also pointed out the difference between the classification effect of the plain Bayesian algorithm and the support vector machine algorithm but did not thoroughly argue the root cause of this difference, which will be the difficulty and the main content of the subsequent research work in this paper.

## Figures and Tables

**Figure 1:** Distribution of pneumonia excluding pneumonia below 60 points.

**Figure 2:** Nonspecific interstitial pneumonia.

**Figure 3:** Desquamative interstitial pneumonia.

**Figure 4:** Lymphocytic interstitial pneumonia, showing a large number of lymphocytes and a small number of plasma cells infiltrating the alveolar septum HE × 100.

**Figure 5:** Generalized interstitial pneumonia.

**Figure 6:** Distribution of pneumonia without excluding pneumonia below 60 points. The horizontal coordinates represent the distribution of interstitial pneumonia, and the vertical coordinates represent the Gaussian density function of the distribution of pneumonia. Test 1 indicates pneumonia in the first test, test 2 indicates pneumonia in the second test, and test 3 indicates pneumonia in the third test.

**Table 1:** Predicted outcomes without excluding pneumonia below 60 points.

	Precision	Recall	*F*l-score	Support
−1	0.89	0.80	0.84	10
1	0.88	1.00	0.93	21
2	0.96	0.92	0.94	26
3	0.94	0.88	0.91	34
4	0.93	0.96	0.94	26
		Accuracy	0.92	117
Macro avg	0.92	0.91	0.91	117
Weighted avg	0.92	0.92	0.92	117

**Table 2:** Predicted outcomes excluding pneumonia with a score below 60.

	Precision	Recall	*F*l-score	Support
1	0.94	1.00	0.97	17
2	1.00	0.96	0.98	26
3	0.90	1.00	0.95	27
4	1.00	0.91	0.95	32
		Accuracy	0.96	102
Macro avg	0.96	0.97	0.96	102
Weighted avg	0.96	0.96	0.96	102

**Table 3:** Pneumonia prediction results using support vector machine algorithm.

	Precision	Recall	*F*l-score	Support
−1	0.91	1.00	0.95	10
1	1.00	0.95	0.98	21
2	1.00	1.00	1.00	26
3	1.00	1.00	1.00	34
4	1.00	1.00	1.00	26
		Accuracy	0.99	117
Macro avg	0.98	0.99	0.99	117
Weighted avg	0.99	0.99	0.99	117

## Data Availability

The datasets used and analyzed during the current study are available from the corresponding author upon reasonable request.
